# Digital Construction of Vocal Music Teaching Resource Base Using Data Mining Technology

**DOI:** 10.1155/2022/8351868

**Published:** 2022-07-30

**Authors:** Ning Xu

**Affiliations:** Liaocheng University Dongchang College, Liaocheng 252000, China

## Abstract

Vocal music teaching resource databases can support teachers' instruction and students' learning while also enhancing the school's ability to run a school because they are the main components of digital construction for vocal music teaching. Currently, system application is the main area of research for DM (data mining), which was previously focused on method discovery. A vocal music teaching resource base based on DM technology is created by using the theme as the central organising principle, processing, and organising the resources. Incorporate lesson planning, teaching, self-study, and output resource construction into a digital network resource application environment by using thematic resource development. Students' achievement data, personal basic information, and evaluation data are used for DM based on the enhanced Apriori algorithm in order to uncover hidden rules and find correlations between various factors. This information is then used to support decision-making. When the system load is 1, the results demonstrate that the Apriori algorithm's CPU waste rate and task success rate is 0.144 and 0.896, respectively. The study's conclusion demonstrates that integrating DM technology into the field of education is theoretically and practically possible and that there is significant room for future study and application in this area.

## 1. Introduction

Traditional vocal music instruction is more abstract because teachers frequently restrict student participation to solo singing and allow them to listen to music tapes in class. A digital information system built on an Internet-connected computer is the vocal music teaching resource database. It uses a computer network as the foundation, treats data as the main component, combines educational materials with information and computer technology, and then produces a shared interactive multimedia vocal music teaching resource database. Teachers can look up relevant reference materials and other relevant information sources for their lesson plans by searching the vocal music teaching resource database. Additionally, students can learn independently by using the Internet to access educational materials at any time and from any location. As a result, we must take advantage of the chance, reevaluate our vocal music education from a fresh perspective, and use cutting-edge computer technology to change the educational model and delivery method.

The formation of beautiful singing is the culmination of the long and ancient art discipline known as vocal music. Data mining (DM) is a technique for obtaining secret forecast data from sizable databases or data warehouses. Machine learning [1, 2], pattern recognition [3, 4], statistics, intelligent databases, knowledge acquisition, data visualisation, high-performance computing, expert systems, and other disciplines are all included in the interdisciplinary field of data mining (DM). The importance of open courseware for global online education was covered by Grunspan et al. in their study of the open courseware and the issues involved. From an economics perspective, this study examines how open educational resources can bring subversive innovation to the field of teaching improvement, but they cannot take the place of traditional school education's economic contribution. It merely serves to support academic instruction. According to Eggink, teachers and students prefer the flipped classroom to the traditional classroom. The flipped classroom method has increased interaction between students and teachers, which has also improved students' interpersonal communication skills. Al-Rasheed and others stressed the necessity of developing a self-expanding teaching resource database system, paying more attention to the free connection and openness of resources, and developing a user-centered resource service system to provide more specialised service features for schools, teachers, and students [5]. Computers are now found in countless households in this quickly evolving information age. People can use the Internet to learn about how the world is changing and developing, and they can use computers to increase the effectiveness and calibre of their work. The use of computers to assist in music instruction has progressively become popular in China's music colleges.

In the field of vocal music teaching, it is full of experience and insight, exploration, and innovation. The construction of a vocal music teaching resource database can integrate excellent digital teaching resources, realize the sharing of teaching resources, and achieve the purpose of improving teaching quality and cultivating professional talents. It can also promote the integration of educational technology and curriculum, and the model provides strong support. Make full use of the audio-visual teaching resource bank to help teachers carry out curriculum reform, stimulate students' learning enthusiasm, constantly broaden learning channels, and finally achieve the greatest educational effect through the audio-visual teaching resource bank. Select typical cases, highlight practical applications, and create modular practice resources. Stimulate and maintain students' interest in learning from various angles, promote the mastery of curriculum knowledge, exercise hands-on ability, and cultivate innovation motivation.

The contributions of this study are as follows. (1) All research is centered on resources, which reflects the effective management and service of the learning process. Well-organized mining and learning resources and effective integration of resources in the process of teaching and learning are two key points and difficulties in current research. Vocal music teaching resource database is an attempt to reconstruct learning resources with the theme as the core and effectively serve the teaching and learning process. (2) According to the construction method and DM technology of the network teaching resource database, a customized retrieval model of the network teaching resource database is established, and the design of the component modules and related algorithms of the model is studied. Establish student submodel, resource submodel, and web access transaction model to model student behavior, teaching resources, and web access, respectively.

## 2. Related Work

### 2.1. DM-Related Research

The meaning of DM refers to the process of extracting potentially useful information and hidden knowledge that people did not know before from a large number of random and fuzzy practical application data. We express the extracted information and knowledge in the form of laws, concepts, patterns, and rules. In DM, it is often used to estimate the fitness of other algorithms, while GA (genetic algorithm) is beneficial to pool data. From the internal relationship between them, useful concepts and patterns can be obtained.

Web information is growing quickly as a result of the development of the Internet. In recent years, the DM field has seen an increase in research on how to efficiently and accurately extract useful information from vast amounts of web data. Wu divides the five application fields of web usage mining into five categories: personality mining, system improvement, site modification, intelligent commerce, and web feature description in accordance with the data source, data type, number of users in the data set, and number of servers in the dataset [6]. The issue of mining association rules among item sets in customer transaction databases was raised by Welte et al., and numerous researchers have since conducted extensive research on this topic [7]. In order to increase the effectiveness of algorithm mining rules and spread the use of association rules, their work includes optimising the original algorithm, such as introducing the concept of random sampling, distributed, and parallel. Many binary tree splitting criteria proofs can be expressed as the weighted sum of two-component drum measure values. This weighted sum method can be used to create two families of split criteria, according to Shao et al. [8]. A hybrid classification algorithm was proposed by Liu et al. that combines the Bayes prior information method with the information gain method of DT (decision tree) classification. It is quicker and more accurate than the Bayes or DT-only classification algorithm [9] when dealing with inconsistent or incomplete data.

Ahn et al. put forward a neural network model combining a rough set with GA, which can simplify the training samples of the network to the greatest extent, optimize the structure of the neural network, and improve the learning efficiency and accuracy of the system. The combination of algorithms has greatly promoted the application of DM classification technology [10]. Danping et al. put forward an algorithm to reduce the dataset to improve the training speed, ensure the classification accuracy, and effectively improve the classification speed [11]. Martinez-Garza et al. proposed a learning algorithm based on a classification and regression tree, which adopted different mobile banking models for customers with different characteristics to improve their security performance [12]. Aifeng et al. used weighted classification roughness as the heuristic function of node selection attribute and proposed a DT construction algorithm based on rough set theory, which is superior to the ID3 algorithm in scale and classification efficiency [13].

### 2.2. Research on Teaching Resource Database

The realization of education informatization needs technical support and information carriers, and the teaching resource database is a collection of various educational resources. It used information technology to integrate education and teaching resources and finally created a shared resource store based on interactive multimedia. A fully functional resource database system should be composed of a teaching resource database, educational resource management system, and network teaching support platform.

Paskins et al. put forward a virtual learning community model, which describes the educational functions of a campus network from seven aspects: communication, teaching, management, resources, extracurricular education, family education, and social education. Among these seven aspects, teaching, school management, and teaching resources are the three most basic aspects of the school [14]. Chen et al. made full use of a large amount of basic data accumulated in the past to make a comprehensive evaluation and decision support for teaching and student management [15]. Özcan Özyurt et al. compared the related contents of DM technology, provided hidden patterns in the database for system managers and decision-makers, excavated potential rules, scientifically evaluated the quality of education and teaching, and provided powerful comprehensive analysis, auxiliary decision-making, and decision-making support services for improving the school's work efficiency, enhancing teaching and scientific research capabilities, drawing up enrollment plans, and training programs [16]. Yu et al. used the DT method and correlation analysis method to analyze the data in the database and found the related factors that affect teaching evaluation and personnel training. The relationships among them, thus providing decision-support information for teaching departments, promote better teaching work and improve teaching quality [17].

Kopcso et al. proposed that based on the concept of the working process and six resource packages, including industry resource package, professional resource package, and curriculum resource package, should be designed for vocal music teaching resource database in secondary vocational schools [18]. It is proposed that the construction of vocal music teaching resource base in secondary vocational schools is explored, and the implementation process is designed from the perspective of school-enterprise cooperation [19]. Zhao proposed that the construction content of the teaching resource database of professional core courses should be divided and constructed from six aspects: electronic lesson plan, multimedia courseware, material database, and test question bank [20].

## 3. Methodology

### 3.1. Construction Method of Vocal Music Teaching Resource Base Based on DM

The vocal music teaching resource bank establishes vocal music teaching tasks, transmits teaching information, imparts knowledge and training skills to students, directly serves students, and has obvious benefits in assisting teaching through database management and network construction. The vocal music teaching resource library offers more options for presenting, storing, editing, and processing all types of educational content. Vocal music majors can simplify teaching challenges, enrich lesson plans, and use flexible teaching techniques. Teachers can easily locate the works they need and allow students to go over them in-depth.

In order to cultivate their ability to appreciate vocal works and allow students to learn from these excellent vocal works flexibly, teachers can teach students a wealth of related knowledge while they are appreciating these vocal works. It can successfully prevent the repeated creation of low-quality resources, maximise the radiation effect of high-quality video teaching resources, and help break the information island of teaching resources into videos. Given that vocal music teaching is a new subject, it is unclear how to build a database of DM practice resources. We planned the DM practice resource bank from two perspectives, content and construction methods, based on extensive research into the construction methods of other related curriculum practice resource banks. The modular design method is used to plan the resources of three layers and four modules in accordance with the usage specifications of various types of resource banks, as shown in Figure 1. In this way, students' enthusiasm for learning vocal music can be sparked by their interest in the subject, inspiring students' strong desire and creativity for musical performance and ultimately enhancing the effectiveness of vocal music instruction.

Based on the existing large-scale teaching resource database, a digital network resource application environment integrating lesson preparation, teaching, self-study, and content resource construction is constructed through the development of special resources. Pay attention to the autonomous learning of subject resources. The online courses and resource application templates automatically generated in the learning process must be interrelated and organically integrated into a whole. The overall architecture of the vocal music teaching resource platform designed in this document is shown in Figure 2.

Teachers use the subject resource curriculum development system and subject resource network classroom system to generate subject resource curriculum and subject online curriculum online and merge them into subject curriculum resources. Extract the subject curriculum template and create the subject resource curriculum, and the subject resource development subsystem generates systematic and organized subject resources. The database teaching platform is not limited by space and time, which can realize the barrier-free learning process, expand and supplement vocal music teaching, and promote the vocal music reform of educational informatization, especially the reform of distance learning mode.

Learning progress query and learning evaluation query: you can inquire about each student's learning situation through the student account, query by grade and student type to know the learning situation of a certain grade or a certain kind of student, and compare them. According to the configuration, multiple log data are used for multiple analyses. Analyze the curriculum structure to help teachers adjust the curriculum structure and teaching content and revise the learning content; The learning behavior evaluation system carries out a variety of evaluations. Teachers evaluate students, students evaluate themselves, and students evaluate students.

Innovative resources are mainly used in course design to guide students to fully apply DM principles and develop DM-based application systems, compilation, preprocessing, algorithm application, result analysis, result interpretation, and presentation, such as DM and image DM. It can also be interdisciplinary, such as the seed selection method for the agriculture and genome clustering algorithm for biology, which fully reflects the application-oriented characteristics of DM. Innovation provides support for cultivating students' innovative consciousness and ability to solve practical problems.

### 3.2. Digital Construction Realization

With the help of personalised service technology, users can receive a variety of services to suit their needs. User data must be gathered and analysed for search engine personalization to understand users' preferences and actions. For the search engine to retrieve information, the user's interest data and search terms are sent to it simultaneously. Offering users services to satisfy their needs for personalised teaching resources in accordance with their behaviours and characteristics is part of a personalised teaching resource service. It contains several specialised services, including UI customization, custom recovery, and custom recommendations.

For an intelligent teaching system, which not only determines the content of the teaching interaction process but also the structure of the learning objectives, domain knowledge representation is crucial. For students in this structure, the system chooses questions and pertinent justifications. Additionally, how knowledge is represented will have an impact on how students' misconceptions are presented. So, using digital multimedia technology, we can accurately recreate that history, let the students personally experience it, and then use singing to discuss the benefits and drawbacks of various musicians so that the students can fully appreciate their inherent differences. A process known as concept-level lifting operation, also known as attribute reduction or attribute generalisation, achieves data generalisation. The same generalised rows can be combined and added in order to reduce the size of the generalised dataset. Users are given access to the results in several different formats, including charts and rulers.

Semantically, the confidence of rules indicates the correctness of rules; the support degree indicates the target percentage that can be deduced from the rule, that is, the importance of the rule to the overall data. Users can define two thresholds, which require that the support and confidence of rules generated by the DM system should not be lower than the given thresholds. The building blocks of the user model perform three functions:

1. Using keywords to create a unique user model from the user personality characteristic library
2. Compile a group user model by identifying the users who share the same interests as the specified users and extracting their features
3. The personalised interest characteristics of the user as well as the interest characteristics of numerous users who share the user's interests are reflected in a comprehensive user model that is created by combining the individual user model and the corresponding group user model

After all the keywords of teaching resources that users are interested in are added to the user's personality database, the comprehensive interest index of keywords must be calculated according to the following formula and filled in the corresponding positions.

(1) $$\begin{array}{c} W_{i}=\left(\frac{D_{t}-D_{i}}{D_{t}-D_{l}}*K\right)+\frac{\left(1-K\right)*C_{i}}{\sum_{h=1}^{400}c_{h}}, \end{array}$$

where *W*_*i*_ is the comprehensive interest index of the keyword *i*, *C*_*i*_, *D*_*i*_ is the cumulative visit times and the latest visit date corresponding to the keyword *i*, *D*_*t*_ is the current date, *D*_*l*_ is the farthest from the current date among all recent access dates, and *K* is the harmonic coefficient, which can be set to 0.7.

To train the classification model, the Bayesian approach is used. The document classification model is discussed in this article, the user's interest and the document's expression align. Assuming that a document's features will all appear separately, *P*(*d|c*_*j*_) can be expressed as the product of conditional probabilities of all features of a document:

(2) $$\begin{array}{c} P\left(d|c_{j}\right)=\prod_{t\in d}p\left(t|c_{j}\right). \end{array}$$

The user's interest archive stores the documents that reflect the user's interest in a certain period to modify the conditional probability corresponding to each category in the vector. Assume that the current action of the user *u* is *a*, its corresponding meaning is *w*_*a*_, the document corresponding to the user action is *d*, and *η* is the learning rate, which is a very small constant. In order to modify the conditional probability associated with each classification in the user interest vector, first, the probability distribution of the document *d* on the classification model must be calculated. The formula is as follows:

(3) $$\begin{array}{c} p\left(t|u\right)\leftarrow \frac{p\left(c_{j}|u\right)+\eta w_{a}p\left(c_{j}|d\right)}{1+\eta w_{a}}. \end{array}$$

Because the business data exist in the data cube of the local memory after preliminary processing and because of the index mechanism of the data cube, it can be searched layer by layer quickly, which improves the execution speed of the algorithm. For the convenience of operation, a new Apriori algorithm implementation method is designed by using a data cube. The algorithm implementation process of the improved Apriori algorithm is shown in Figure 3.

The specific steps are as follows:

1. Establish a transaction data table, which converts students' achievement data for two courses into Boolean representation
2. Call the stored procedure, count the occurrence times of each item, and store it in the data table of the frequent item set
3. The deletion support count is less than the minimum support, and all frequent item sets are taken out. If the number of candidate item sets is found to be zero, the operation stops the output of frequent item sets of all elements. The number of times the program scans the transaction data table depends on the maximum length of frequent item sets.
4. Calculate the confidence of each nonempty subset of the final frequent item sets, delete the records less than the minimum confidence threshold, and finally generate rules and store them in the data table

According to the methods and rules of attribute *A* analysis, it is necessary to screen the achievement attribute information and adopt two methods: attribute generalisation and attribute elimination. The information gained by dividing the sample set of the current branch node by using the attribute is

(4) $$\begin{array}{c} \text{Gain}\left(A\right)=I\left(S_{1},\ldots ,S_{m}\right)-E\left(A\right). \end{array}$$

This function is the core function in the DT algorithm, and it is the basis for selecting node attributes. Calculate Info according to the formula of information theory:

(5) $$\begin{array}{c} \text{Info}\left(S\right)=\text{Info }\left(S_{p},S_{n}\right)=-\left(\frac{x}{x+y}\log\frac{x}{x+y}+\frac{y}{x+y}\log\frac{y}{x+y}\right). \end{array}$$

Calculate the information entropy according to the above formula:

(6) $$\begin{array}{c} E\left(A\right)=\sum_{j=1}^{v}\frac{S_{1j}+S_{2j}+\cdots +S_{mj}}{S}I\left(S_{1j},\ldots ,S_{mj}\right). \end{array}$$

The former part of data is the error obtained by idealized classification, that is, impure, while the latter part of the data is the actual error obtained if a certain attribute is used for classification, and the value obtained after making a difference is the variation of impure.

Under the current system, we mainly consider three aspects in evaluating students' cognitive ability: memory, understanding, and application. In order to objectively evaluate students' abilities in three aspects, the learning test method is adopted. In the test questions, the weight levels of memory, understanding, and application corresponding to each question are set. These levels are given by teaching experts according to the knowledge points examined in the test questions. Use the following formula to calculate each cognitive ability score.

(7) $$\begin{array}{c} A_{j}=\frac{\sum_{i=1}^{m}t_{i}\cdot r_{ij}}{\sum_{i=1}^{m}r_{ij}}. \end{array}$$

Teachers' evaluation of students is fuzzy, and the evaluation results are fuzzified. Fuzzy the students' cognitive ability into three levels, namely, *P*={low,middle,high}. Finally, the DT shown in Figure 4 is generated.

Because the processing of data files in local space does not need transmission time, it can be processed directly, so it can exchange processing time by storing some copies. So, the time to complete a job is the sum of file transfer time and file processing time:

(8) $$\begin{array}{c} T_{{\text{homework}}_{i}}=\sum T_{\text{transmit}}+\sum T_{\text{document}}. \end{array}$$

Therefore, for jobs submitted by all users, the total processing time is

(9) $$\begin{array}{c} T_{\text{total time}}=\sum T_{{\text{homework}}_{i}}. \end{array}$$

The above is the process of DT learning of teaching methods. If all teaching strategies are DT-learned, the system will be able to find out what kind of students are suitable for adopting what kind of teaching strategies, and the intelligence of the system will be improved accordingly.

## 4. Experiment and Results

We select the database of students' personal basic information and the database of students' scores with relatively complete information items as experimental objects and intercept the basic information and scores of vocal music students as training sets to verify the system. We take the relationship between gender, native place, admission method, major before admission, and whether the score of a vocal music course is *A* as an example to verify the feasibility and correctness of the system. If minsup=1 and minconf=10 are preset, the rule set shown in Figure 5 can be obtained again.

Although not all strong association rules for the experimental data obtained have practical guiding significance, the information they contain can still be useful for decision-making when analysing their data, particularly when analysing the changes of strong association rules under various support and confidence thresholds. It is clear that the vocal music course strongly depends on whether students are working on computers. It is challenging to succeed in this course to a high level without long-term computer literacy. On the other hand, if we examine how our undergraduate experiences affected how well, we performed in our vocal music classes, we can say that there was little to no difference. We use the direct data transmission method rather than the fusion optimization method as the reference object of the experiment in order to compare the effects of the cache synchronization algorithm based on transaction merge optimization on communication data volume, communication cost, synchronization time, and conflict.  Figure 6 shows the execution time of the synchronization algorithm, which is one of the key metrics used to assess the algorithm's quality.

It can be seen that because the record merging optimization algorithm directly merges the cached records locally and streams them and the remote pull statement directly updates the database, the processing speed is faster, so the synchronization time is basically faster than the traditional one. The acquisition speed of data remote updates will also slow down, so the time base is relatively large at first and then increases linearly with the increase of disconnection time. The number of conflicts refers to the number of transaction submission errors caused by conflicts. As can be seen from Figure 7, the system synchronization algorithm is executed according to the time stamp, which basically does not happen. Original methods usually update bad tuples after synchronization and as the number of end clients increases.

It can be seen that the synchronization algorithm optimized by semantic-based transaction merging can effectively reduce the amount of data transmitted synchronously, the execution time of the synchronization algorithm, and the number of tuples with update errors. The number of conflicts will gradually emerge. Therefore, the data synchronization algorithm model based on semantic transaction merging optimization provides a feasible solution for mobile database synchronization. Use grid technology to select rendering sites for work and select replacement copies for each site. Consider using grid technology to select a processing site for the job and copy replacement for each site. Considering that all sites can keep copies of files, when the storage capacity is insufficient, files can be deleted appropriately according to the algorithm. The results are given in Table 1.

Due to the evaluation of different workloads, we can draw the following conclusions from the experimental data: without the existing spatial database, the average running time becomes unstable and takes a long time, the network utilization rate is high, and the storage utilization rate is low. The algorithm limits the counting period to a specific time interval, but it does not strictly reflect the recent visits. Therefore, while deleting files, some useful files may also be deleted, so when the workload increases, there is no obvious change in network utilization.

The processing performance of spatial jobs in grid environment is far superior to the existing spatial database system because the reasonable file replacement algorithm in grid environment wins high-performance job processing for job processing in grid environment, which can reduce the utilization rate of network resources and improve the utilization rate of storage resources. In the grid spatial database model, in order to verify the impact of each grid resource allocation and scheduling algorithm on the overall performance, we assume that the grid spatial database scenario is fixed. We introduce the use of computing units as evaluation parameters. The utilization rate of computing units under different workloads is shown in Figure 8.

For a random algorithm, the utilization rate of spatial data processing units is the lowest and the average operation time is the highest due to the random selection of spatial data processing units, which causes instability in key metrics like queue length and processing time. The queue length algorithm can balance the length of the queue among the units that process spatial data, but the processing time varies because different spatial jobs have different working hours. The access cost integration algorithm can take into account how long each spatial data processing unit actually runs, forming a load balance between them. This is due to the fact that the coordination of various spatial data processing resources results in performance that improves with increasing workload by fully taking into account the queue length as the result of two factors and processing time.

Figure 9 shows the influence of the Apriori algorithm on CPU time waste rate and main task success rate of the system. Because the Apriori algorithm tries to avoid preempting low-priority tasks that are about to be completed and take a long time to execute, it can effectively reduce the CPU time waste, thus reducing the CPU waste rate of the whole system. The CPU waste rate and task success rate of the Apriori algorithm are 0.144 and 0.896, respectively, when the system load is 1. The replacement task time of the low-priority task released later can be used by other main tasks, which increases the success probability of other main tasks, thus improving the task success rate of the whole system.

In this study, the questionnaire was used to complete the systematic evaluation. Ten questions were designed from three aspects, complete system, resource application, and interactive community, and were investigated in some vocal vocational courses. The theme courses generated by this system should not be simply equivalent to theme websites, thematic websites, or online courses, but should have their unique designs in theme setting, resource application, and interactive community design. The evaluation results are given in Table 2.

The survey results show that the majority of college teachers and students give a high evaluation of this system, and the vast majority of respondents think that this system can well meet the needs of the new curriculum reform for college vocal music teaching and can play an effective role. To meet the needs of university professors and in order to meet the needs of students for learning discipline resources, most university professors and administrators believe that the system can fully support the development of research-based learning in universities. Using this system makes the subject course simple, convenient, and easy to learn, and the generated subject course has clear structure, reasonable logic, and high technical content. It has a high practical application value and can play an important supporting role in teachers' information teaching design and information classroom teaching.

## 5. Conclusions

The creation of a database of resources for university-level vocal music instruction is an organized, protracted project that requires the involvement and support of both teachers and students. This study makes a first attempt at the overall DM process to address this issue. The preliminary findings demonstrate that it is theoretically and practically possible to use DM technology for the digital construction of vocal music instruction. Create the corresponding vocal music teaching resource database, give teachers access to a potent information-based teaching design and research platform, create a vibrant student interest group platform, enhance teacher-student interaction, and create a system for communicating between homes and schools in order to fully realize the concept of a people-oriented educational system. This system pays close attention to comprehending the laws of education and teaching, fully considers the characteristics of teachers' teaching, and applies it to the system's reasoning rules, reflecting the dominant role of educational ideas and theories and combining the characteristics of teachers' teaching. Increase the specificity and diversity of vocal music instruction, support Chinese vocal music students' capacity for independent study, and offer a fresh opportunity for the advancement of vocal music art in China.

## Figures and Tables

**Figure 1:** Functional design.

**Figure 2:** The overall structure of vocal music teaching resource database platform.

**Figure 3:** Algorithm realization process of the Apriori algorithm.

**Figure 4:** Generated DT of training.

**Figure 5:** Generated rule set.

**Figure 6:** Synchronization algorithm execution time.

**Figure 7:** Conflicts of transactions.

**Figure 8:** Different workload of algorithms and utilization ratio of spatial data processing units.

**Figure 9:** The influence of Apriori on CPU waste rate and task success rate.

**Table 1:** Simulation data of grid space database based on the optimization algorithm.

Space workload	Storage unit utilization rate (%)	Average operation time (s)	Network utilization rate (%)
100	63.2	81.4	82.2
500	63.2	79.9	75.6
1000	63.2	79.6	75.9
1500	63.2	80.1	64.3

**Table 2:** The evaluation of theme courses.

Project	Aggregate score	Score
Knowledge processing	63.2	59.1
Content organization	33.1	28.6
Technical level	9.8	9.1

## Data Availability

The data used to support the findings of this study are available from the corresponding author upon request.
